This article has been retracted.

# Effect of EPOC on Serum MicroRNA Expression in Patients with Hypertension

**DOI:** 10.1155/2022/1998445

**Published:** 2022-02-23

**Authors:** Hao Li

**Affiliations:** Physical Education Department of North Sichuan Medical College, 55 Dongshun Road, Gaoping, Nanchong, Sichuan 637100, China

## Abstract

In order to analyze the effect of EPOC on serum microRNA expression in patients with hypertension, we have carried out an experimental evaluation and presented a dedicated method to improve its effectiveness. For this purpose, 60 patients with hypertension treated in our hospital from January to December 2020 were selected and randomly divided into the EPOC group (30 cases) and the control group (30 cases). Patients in both groups received conventional hypertension medication according to the treatment guidelines, and education and guidance were strengthened to ensure patients' drug compliance. The EPOC group received EPOC training in addition to conventional medication. After the intervention, 6MWD, LVEF, and LVEDD in the control group and the EPOC group were significantly improved compared with that before treatment (*P* < 0.05). The improvement of cardiac function in the EPOC group was significantly better than that in the control group (*P* < 0.05). Physiological function, physiological characteristics, body pain, and general health of the control group and the EPOC group were significantly improved compared with that before treatment (*P* < 0.05). The improvement of quality of life in the EPOC group was significantly better than that in the control group (*P* < 0.05). The indexes of heart rate, oxygen pulse, minute ventilation, oxygen uptake in kg, and anaerobic threshold in the EPOC group were significantly better than those in the control group before and after treatment (*P* < 0.05). Full-sample real-time PCR verification of the 8 miRNAs with the highest expression differentiation showed that, compared with the control group, the expression levels of miR-20a-5p, miR-93-5p, and miR-1287-5p in the serum of the EPOC group were significantly increased, while the expression levels of miR-7706, miR-28-5p, and miR-125b-5p were significantly decreased. The expression of miR-20a-5p was the highest, while the expression of miR-125b-5p was the lowest, suggesting that miR-20a-5p and miR-125b-5p might be involved in the process of HIIT to improve hypertension. After EPOC rehabilitation treatment, patients' heart function indexes, lung function indexes, and quality of life have been significantly improved. EPOC rehabilitation can improve exercise tolerance, enhance cardiopulmonary function, and improve the prognosis of patients.

## 1. Introduction

Hypertension can cause myocardial damage characterized by fibrillation of blood vessels and tissue spaces, leading to hardening of the cardiac tissue and heart failure. In recent years, with the increasing incidence and mortality of cardiovascular diseases, the prevention and treatment of myocardial fibrosis are of great significance to control the development of hypertensive heart damage and improve the prognosis of the disease [1, 2]. Human microRNAs (miRNAs) are noncoding RNAs, and current studies have shown that a variety of RNAs are closely related to cardiovascular diseases [3]; it is widely expressed in the cardiovascular system and plays an important role in physiological regulation, especially in the pathological process of hypertension [4]. However, preliminary studies have confirmed that regular exercise can significantly regulate the expression profile of serum miRNA [5]. Clinical practice has proved that exercise rehabilitation is an effective way to treat hypertension, which can significantly reduce the recurrence, delay the progression of the disease, and reduce the incidence of adverse cardiac events. It is an extremely important second-level prevention strategy [6]. Excess postexercise oxygen consumption (EPOC) is a kind of exercise that can give full, rapid, and concentrated exercise in a short time. Although most muscles stop exercising after exercise, the oxygen intake does not return to the quiet state before exercise because the energy metabolism does not return to the quiet state before exercise [7]. At present, foreign studies have confirmed that EPOC training for 8 consecutive weeks is safe and effective for patients with hypertension, and its effect is better than that of the traditional regular aerobic exercise [8]; however, there are few reports on the molecular regulation mechanism of the pathophysiological effects of hypertension. Therefore, this study will explore the rehabilitation effect of EPOC training on patients with hypertension and the relevant mechanism of microRNA participating in exercise benefit in hypertension prevention.

In order to analyze the effect of EPOC on serum microRNA expression in patients with hypertension, we have carried out an experimental evaluation and presented a dedicated method to improve its effectiveness. For this purpose, 60 patients with hypertension treated in our hospital from January to December 2020 were selected and randomly divided into the EPOC group (30 cases) and the control group (30 cases). Patients in both groups received conventional hypertension medication according to the treatment guidelines, and education and guidance were strengthened to ensure patients' drug compliance. The EPOC group received EPOC training in addition to conventional medication. After the intervention, 6MWD, LVEF, and LVEDD in the control group and the EPOC group were significantly improved compared with that before treatment (*P* < 0.05). The improvement of cardiac function in the EPOC group was significantly better than that in the control group (*P* < 0.05). Physiological function, physiological characteristics, body pain, and general health of the control group and the EPOC group were significantly improved compared with that before treatment (*P* < 0.05).

The rest of the paper is organized as given as follows. In the subsequent section, the proposed methodology that is improving the effectiveness of the proposed methodology is described in detail. Experimental results and observations were presented in the subsequent section in both textual and graphical or tabular forms. A generalized discussion section is provided to provide a brief description of the problem at hand, the proposed solution, and its effectiveness. Finally, concluding remarks along with future directives are presented along with reference materials.

## 2. Proposed Methodology

### 2.1. General Information

60 patients with hypertension treated in our hospital from January to December 2020 were selected and randomly divided into the EPOC group (30 cases) and the control group (30 cases). All patients signed the ethical informed consent letter. There was no statistical difference in baseline data between the two groups (*P* > 0.05).

#### 2.1.1. Inclusion Criteria

Inclusion criteria were defined as follows:

1. Age 18∼75 years old
2. First diagnosed as hypertension and no medication was taken
3. Met the diagnostic criteria of the “Chinese Guidelines for the Prevention and Treatment of Hypertension (2010 Revised Edition)” [9]
4. Those who had high compliance with sports rehabilitation and could complete 8 weeks of training
5. Irregular exercise history (exercise 2-3 times a week, more than 30 min each time)

#### 2.1.2. Exclusion Criteria

Exclusion criteria were defined as follows:

1. Secondary hypertension, or with liver, kidney, lung, and other organ system fibrous lesions
2. Arrhythmia with hemodynamic abnormalities
3. Coronary heart disease, acromegaly, or diabetes
4. Asthma, COPD, pulmonary embolism, and stroke which makes unable to carry out high-intensity exercise
5. Arthritis, rheumatism, rheumatism, or other orthopedic diseases caused the inability to train normally
6. Patients with doctor-patient communication barriers
7. Others who believed that sports training was not possible

General information is shown in Table 1.

### 2.2. Methodology

Patients in both groups received conventional hypertension medication according to the treatment guidelines, and education and guidance were strengthened to ensure patients' drug compliance.

#### 2.2.1. EPOC Group

In addition to conventional medication, patients received EPOC training as follows: 75%∼80% HRmax training 4 min + 50% HRmax recovery 3 min; there were 4 groups of training, a total of 28 min, warm-up for 5 min before training and relax for 5 min after training 4 times/week for 8 weeks. All the training was carried out under supervision. Patients' heart rate, blood pressure, and subjective tiredness were closely monitored. If they felt unwell, they should stop exercising immediately [10]. Cardiopulmonary exercise test and heart color ultrasound were performed before training to evaluate patients' cardiac function, exercise ability, and fatigue grade. After 8 weeks of training, a cardiopulmonary exercise test was performed again.

### 2.3. Observational Index

#### 2.3.1. Cardiac Function

6 min walking distance (6MWD), left ventricular ejection fraction (LVEF), and left ventricular end-diastolic diameter (LVEDD) were recorded before and after intervention in 2 groups.

#### 2.3.2. Quality of Life

A 36-item concise health status questionnaire (SF-36) [11] was used to evaluate the quality of life of each group at the time of enrollment and the follow-up visit at the end of treatment.

#### 2.3.3. Assessment of Lung Function and Exercise Tolerance

The indexes of lung function and exercise tolerance, including heart rate, oxygen pulse (O2/HR), minute ventilation, oxygen uptake in kg (VO_2_/kg), and anaerobic threshold (AT), were detected by Keshi Mai cardiopulmonary exercise assessment instrument [12].

#### 2.3.4. MicroRNA Gene Analysis and Real-Time PCR Verification and Quantitative Determination

At the time of enrollment, 5 mL of elbow venous blood was collected from all subjects and placed in an EDTA tube. The plasma was separated by centrifugation at 20 000 r/min at 4°C for 10 min, the supernatant was transferred, and repeated centrifugation was performed to remove impurities. High-throughput analysis of the microRNA microarray (Affymetrix GeneChip miRNA 4.0, Affymetrix, USA) was performed [13], and data statistics and hierarchical cluster analysis were performed using the analysis software provided by the chip company. The total miRNA in serum was isolated and extracted using the Ambion mirVana miRNA Isolation Kit (Thermo Fisher, USA), and then, the total miRNA extracted was retrotranscribed using the reverse transcription kit to obtain the corresponding cDNA chain of the miRNA. Then, fluorescence quantitative detection of the whole sample miRNA was performed. U6 was used as the internal reference gene, and the relative expression level of the target miRNA was calculated using the 2^−ΔΔ*Ct*^ method. The reaction parameters of C1000 touch gradient PCR were 94 °C for 20s and 60 °C for 34s, a total of 40 cycles. The experimental operation was carried out according to the instructions of the kit. Primer sequences are shown in Table 2.

### 2.4. Statistical Method

All data were analyzed by SPSS 22.0 statistical software. Measurement data were expressed as mean ± standard deviation (*x* ± *s*). *t*-test was used to compare the differences between groups, and paired *t*-test was used for intragroup comparison before and after treatment. Enumeration data were expressed by case number (constituent ratio), and *χ*^2^ test was used for comparison between groups. *PP* < 0.05 was considered statistically significant.

## 3. Experimental Results

### 3.1. Results of Cardiac Function

Before the intervention, there was no significant difference in cardiac function indexes between the control group and the EPOC group (*P* > 0.05). After the intervention, 6MWD, LVEF, and LVEDD in the control group and the EPOC group were significantly improved compared with that before treatment (*P* < 0.05). The improvement of cardiac function in the EPOC group was significantly better than that in the control group (*P* < 0.05), and it was suggested that EPOC could improve the cardiac function of patients with hypertension and promote their recovery. Results of cardiac function are shown in Table 3.

### 3.2. Results of Quality of Life

Before the intervention, there was no significant difference in the quality of life indexes between the control group and the EPOC group (*P* > 0.05). After the intervention, physiological function, physiological characteristics, body pain, and general health of the control group and the EPOC group were significantly improved compared with that before treatment (*P* < 0.05). The improvement of quality of life in the EPOC group was significantly better than that in the control group (*P* < 0.05), and it was suggested that EPOC would help improve the quality of life of patients with hypertension. Results of quality of life are shown in Table 4.

### 3.3. Results of Assessment of Lung Function and Exercise Tolerance

Before the intervention, there was no significant difference in lung function between the control group and the EPOC group (*P* > 0.05). After the intervention, the indexes of heart rate, oxygen pulse, minute ventilation, oxygen uptake in kg, and anaerobic threshold in the EPOC group were significantly better than those in the control group before and after treatment (*P* < 0.05). It was suggested that EPOC could improve lung function and exercise tolerance in patients with hypertension. Results of the assessment of lung function and exercise tolerance are shown in Table 5.

### 3.4. Results of miRNA Expression

The differences in miRNA expression profiles between the control group and the EPOC group after the intervention were detected by the Affymetrix GeneChip miRNA chip, which covered 30430 probe groups of mature miRNAs and 2014 human miRNA precursors. The screening standard of differential genes was Q-value ≤5%. Through miRNA microarray screening, 91 genes were differentially expressed. Full-sample real-time PCR verification of the 8 miRNAs with the highest expression differentiation showed that, compared with the control group, the expression levels of miR-20a-5p, miR-93-5p, and miR-1287-5p in the serum of the EPOC group were significantly increased, while the expression levels of miR-7706, miR-28-5p, and miR-125b-5p were significantly decreased. The expression of miR-20a-5p was the highest, while the expression of miR-125b-5p was the lowest, suggesting that miR-20a-5p and miR-125b-5p might be involved in the process of EPOC to improve hypertension.

## 4. Discussion

Under the common influence of social aging, living habits, and environmental pollution, the prevalence of hypertension in the Chinese population has increased significantly. Hypertension is essentially an ischemic cardiovascular disease [14]. Clinical practice has long proved that exercise rehabilitation is an important auxiliary means in the treatment of hypertension. Combined with drug management, risk factor control, and a good lifestyle, it can significantly reduce the occurrence of cardiovascular events and sudden death, and exercise rehabilitation has become an important content of hypertension treatment research [15, 16]. However, the mechanism of excess oxygen consumption after exercise is still not clear. Some scholars believe that the influence of excess oxygen consumption after exercise is mainly based on exercise intensity. At the same time, whether excessive oxygen consumption after high-intensity exercise is the main cause of large amount of fat oxidation still needs further study. It is necessary to carry out tracking detection of oxygen intake after exercise for 24∼48 h, even to detect the oxygen intake under the quiet state, and determine the total amount of excessive oxygen consumption and fat oxidation after exercise [17]. Compared with traditional aerobic exercise, EPOC can enhance people's aerobic capacity and exercise tolerance and improve cardiopulmonary function. Wu Guangsheng found that EPOC could effectively improve the levels of fasting blood glucose and 2 h postprandial blood glucose in patients with prediabetes, and the effect of reducing fat was better than that of traditional moderate-intensity sustained exercise [18]. Studies have shown that EPOC is better than moderate exercise, which can improve the exercise endurance and cardiopulmonary function of patients with coronary diseases. In addition, safety evaluations of several studies have shown that high-intensity aerobic interval exercise under the guidance of a professional rehabilitation physician does not increase the incidence of adverse cardiovascular events in patients with hypertension [19]. However, at present, there is no research report about the effect of EPOC on hypertension patients in China [20].

The results of this study showed that after the intervention, 6MWD, LVEF, and LVEDD in the control group and the EPOC group were significantly improved compared with that before treatment (*P* < 0.05). The improvement of cardiac function in the EPOC group was significantly better than that in the control group (*P* < 0.05) Physiological function, physiological characteristics, body pain, and general health of the control group and the EPOC group were significantly improved compared with that before treatment (*P* < 0.05). The improvement of quality of life in the EPOC group was significantly better than that in the control group (*P* < 0.05). The indexes of heart rate, oxygen pulse, minute ventilation, oxygen uptake in kg, and anaerobic threshold in the EPOC group were significantly better than those in the control group before and after treatment (*P* < 0.05). Full-sample real-time PCR verification of the 8 miRNAs with the highest expression differentiation showed that, compared with the control group, the expression levels of miR-20a-5p, miR-93-5p, and miR-1287-5p in the serum of the EPOC group were significantly increased, while the expression levels of miR-7706, miR-28-5p, and miR-125b-5p were significantly decreased. The expression of miR-20a-5p was the highest, while the expression of miR-125b-5p was the lowest, suggesting that miR-20a-5p and miR-125b-5p might be involved in the process of HIIT to improve hypertension.

## 5. Conclusion

In order to analyze the effect of EPOC on serum microRNA expression in patients with hypertension, we have carried out an experimental evaluation and presented a dedicated method to improve its effectiveness. For this purpose, 60 patients with hypertension treated in our hospital from January to December 2020 were selected and randomly divided into the EPOC group (30 cases) and the control group (30 cases). Patients in both groups received conventional hypertension medication according to the treatment guidelines, and education and guidance were strengthened to ensure patients' drug compliance. The EPOC group received EPOC training in addition to conventional medication. After the intervention, 6MWD, LVEF, and LVEDD in the control group and the EPOC group were significantly improved compared with that before treatment (*P* < 0.05). The improvement of cardiac function in the EPOC group was significantly better than that in the control group (*P* < 0.05). Physiological function, physiological characteristics, body pain, and general health of the control group and the EPOC group were significantly improved compared with that before treatment (*P* < 0.05). In conclusion, after EPOC rehabilitation treatment, patients' heart function indexes, lung function indexes, and quality of life have been significantly improved. EPOC rehabilitation can improve exercise tolerance, enhance cardiopulmonary function, and improve the prognosis of patients.

## Figures and Tables

**Table 1:** General information.

General information		EPOC group	Control group	*P*
Cases		30	30	＞0.05
Gender (*n*)	Male	17	18	＞0.05
	Female	13	12	
Age (average)		46.28 ± 9.24	45.61 ± 8.33	＞0.05
BMI (kg/m^2^)		22.07 ± 3.18	23.14 ± 2.69	＞0.05
Diabetes (*n*)		15	13	＞0.05
Hyperlipidaemia (*n*)		11	10	＞0.05

**Table 2:** Primer sequences.

Primers	q RT-PCR forward: (5′-3′)	q RT-PCR reverse (5′-3′)
U6	GTCGGTACAGATCTGTGGCAC	GATTATCGGCCCCGCGACATTC
miR-20a-5p	CTTATGCCATCTT GGCGG	CGCGTACCGGAGT CAGG
miR-28-5p	CATCCGGAGAGACGGACAT	TTGTACAGCTGCAGTGGAC
miR-93-5p	GTCCAGGTGAGAGTGTCGT	GGTCATGTGCTACGTTT
miR-125b-5p	GGGCAGAGGGC GGATT	AGGATCAGT GCTAC
miR-1287-5p	CTGAGGGCA GGGACATCGT	GGTCTTCATCGCGAGGGCGG
miR-7706	TTCGAGAAGTGCAG CGAC	AGTACTCGCCGATTGTGGC

**Table 3:** Results of cardiac function.

Groups		EPOC group	Control group	*P*
6MWD	Before intervention	339.25 ± 15.33	341.52 ± 12.58	>0.05
	After intervention	426.72 ± 12.81	380.44 ± 11.69	<0.05

LVEF	Before intervention	51.46 ± 4.98	53.29 ± 5.01	>0.05
	After intervention	66.98 ± 6.12	59.36 ± 6.07	<0.05

LVEDD	Before intervention	57.15 ± 5.36	58.05 ± 4.94	>0.05
	After intervention	46.48 ± 3.62	51.27 ± 4.03	<0.05

**Table 4:** Results of quality of life.

Groups		EPOC group	Control group	*P*
Physiological function	Before intervention	73.24 ± 6.47	73.02 ± 8.15	>0.05
	After intervention	83.95 ± 7.12	78.12 ± 6.69	<0.05

Physiological characteristics	Before intervention	34.82 ± 3.64	38.44 ± 4.15	>0.05
	After intervention	68.95 ± 7.59	51.01 ± 5.17	<0.05

Body pain	Before intervention	52.43 ± 6.54	50.04 ± 5.59	>0.05
	After intervention	72.89 ± 8.04	66.24 ± 4.27	<0.05

General health	Before intervention	40.78 ± 5.29	41.09 ± 5.04	>0.05
	After intervention	69.81 ± 7.65	51.33 ± 6.28	<0.05

**Table 5:** Results of the assessment of lung function and exercise tolerance.

Groups		EPOC group	Control group	*P*
Heart rate	Before intervention	72.25 ± 8.05	71.53 ± 7.64	>0.05
	After intervention	108.99 ± 15.41	102.18 ± 15.44	<0.05

Oxygen pulse	Before intervention	10.78 ± 1.38	11.20 ± 1.05	>0.05
	After intervention	12.68 ± 2.47	11.74 ± 1.62	<0.05

Minute ventilation	Before intervention	36.15 ± 7.09	36.40 ± 8.14	>0.05
	After intervention	43.59 ± 6.78	37.28 ± 8.06	<0.05

Oxygen uptake in kg	Before intervention	50.16 ± 14.22	52.27 ± 17.06	>0.05
	After intervention	68.15 ± 19.30	53.09 ± 15.14	<0.05

Anaerobic threshold	Before intervention	46.35 ± 1.05	45.88 ± 1.87	>0.05
	After intervention	61.27 ± 3.24	49.15 ± 3.41	<0.05

## Data Availability

The data used to support the findings of this study are included within the article.

## References

[1] Ni L., Xue P., An C. (2021). Establishment of normal range for thromboelastography in healthy middle-aged and elderly people of Weihai in China. *Journal of Healthcare Engineering*.

[2] Zheng L., Feng H., Yin L. (2021). Study on the correlation factors of tumour prognosis after intravascular interventional therapy. *Journal of Healthcare Engineering*.

[3] Tian J., An X., Niu L. (2017). Role of microRNAs in cardiac develop-ment and disease. *Experimental and Therapeutic Medicine*.

[4] Ding X.-Q., Ge P.-C., Liu Z. (2015). Interaction between microRNA expression and classical risk factors in the risk of coronary heart disease. *Scientific Reports*.

[5] ’Souza R. F., Woodhead J. S. T., Zeng N. (2018). Circulatory exosomal miRNA following intense exercise is unrelated to muscle and plasma miRNA abundances. *American Journal of PhysiologyEndocrinology and Metabolism*.

[6] Srikanth S., Deedwania P. (2016). Management of dyslipidemia in patients with hypertension, diabetes, and metabolic syndrome. *Current Hypertension Reports*.

[7] Wang R. (2002). *Exercise physiology*.

[8] Moholdt T. T., Amundsen B. H., Rustad L. A. (2009). Aerobic interval training versus continuous moderate exercise after coronary artery bypass surgery: a randomized study of cardiovascular effects and quality of life. *American Heart Journal*.

[9] Sun G. (2011). Interpretation of the updated content of “guidelines for prevention and treatment of hypertension in China (2010 revised edition)”. *Tianjin Medical*.

[10] Yang W., Shao H., Cao Y. (2016). Analysis of microRNA expression profile in patients with hypertensive intracerebral hemorrhage. *World Traditional Chinese Medicine*.

[11] Nakao M., Yamauchi K., Ishihara Y., Solongo B., Ichinnorov D., Breugelmans R. (2016). Validation of the Mongolian version of the SF-36v2 questionnaire for health status assessment of Mongolian adults. *SpringerPlus*.

[12] Yuan F., Wang Y., Liu K., Kong H., Xie W. (2021). The significance of cardiopulmonary exercise test in the diagnosis and treatment of pulmonary hypertension. *International Respiratory Journal*.

[13] Mccall M. N., Murakami P. N., Lukk M., Huber W., Irizarry R. A. (2011). Assessing affymetrix GeneChip microarray quality. *BMC Bioinformatics*.

[14] Luo X. (2016). Discussion on the rising incidence of hypertension from common cases. *Chinese Journal of Hypertension*.

[15] Mackenzie A., Johnson M. (2015). Demand for exercise training in patients with pulmonary arterial hypertension in Scotland. *European Respiratory Journal*.

[16] Babu A. S., Padmakumar R., Maiya A. G. (2013). A review of ongoing trials in exercise based rehabilitation for pulmonary arterial hypertension. *Indian Journal of Medical Research*.

[17] Dong X., Chen Y., Han J. (2016). Substrate metabolism and energy consumption characteristics based on different body weights and exercise methods. *Chinese Journal of Sports Medicine*.

[18] Neto A., Silva N., Farinatti P. (2015). Influence of resistance training variables on excess postexercise oxygen consumption: a systematic review. *Revista Brasileira de Medicina do Esporte*.

[19] Oparil S., Giles T., Ofili E. O. (2011). Moderate versus intensive treatment of hypertension with amlodipine/valsartan for patients uncontrolled on angiotensin receptor blocker monotherapy. *Journal of Hypertension*.

[20] Leggio M., Mazza A., Cruciani G. (2014). Effects of exercise training on systo-diastolic ventricular dysfunction in patients with hypertension: an echocardiographic study with tissue velocity and strain imaging evaluation. *Hypertension Research*.

